# Study on the Risk Factors of Pulmonary Infection after Laparoscopic Surgery and Analysis of the Detection Results of Drug-Resistant Bacteria

**DOI:** 10.1155/2022/6510068

**Published:** 2022-03-18

**Authors:** Tingting Zhai, Liwei Zhang, Jing Sun, Yuanchun Li, Jie Hou, Fengxia Du

**Affiliations:** ^1^Nursing Department, The Second Affiliated Hospital of Qiqihar Medical University, Qiqihar 161000, China; ^2^Department of Gastroenterology, The Second Affiliated Hospital of Qiqihar Medical University, Qiqihar 161000, China; ^3^Department of General Surgery, The Second Affiliated Hospital of Qiqihar Medical University, Qiqihar 161000, China; ^4^Operating Room, The Fourth Affiliated Hospital of Harbin Medical University, Harbin 150000, China; ^5^Department of Etiology, Qiqihar Medical University, Qiqihar 161000, China

## Abstract

This study aimed to investigate and analyze the risk of pulmonary infection after laparoscopic surgery and the detection results of drug-resistant bacteria. With the laparoscopic technology developing rapidly in recent years and people's minimally invasive concept improving continuously, laparoscopic radical surgery has been widely used in the treatment of a variety of diseases. Laparoscopic surgery has the probability of causing complications. In order to avoid this, the risk factors after surgery were analyzed, and the drug-resistant bacteria were analyzed for accurate prevention and treatment. A total of 600 patients who underwent elective laparoscopic surgery in our hospital from January 2017 to September 2021 were included in the study. The risk factors and pathogen distribution of pulmonary infection were analyzed. The risk factors of pulmonary infection after laparoscopic surgery were hypoproteinemia, diabetes mellitus, pulmonary disease history, and perioperative blood transfusion. The main pathogens were *Klebsiella pneumoniae*, *Staphylococcus aureus*, *Pseudomonas aeruginosa*, *Escherichia coli*, and *Streptococcus pneumoniae*. In clinical work, relevant nursing intervention measures can be developed for the above factors, so as to reduce the incidence of pulmonary infection. This study finds the risk factors for pulmonary infection after surgery, and the common drug-resistant bacteria has an indicative and guiding effect on the formulation of nursing management measures.

## 1. Introduction

With the laparoscopic technology developing rapidly in recent years and people's minimally invasive concept improving continuously, laparoscopic radical surgery has been widely used in the treatment of a variety of diseases. Compared with traditional open surgery, it has advantages such as less trauma, less patient pain, and faster postoperative recovery [1]. However, laparoscopic surgery is still one of the invasive operations, which may also cause a series of surgical complications, including incision infection, lung infection, urinary tract infection, and catheter-related infection [2, 3]. After exploring relevant reports abroad, more detailed conclusions can be drawn, which also plays an important role in the knowledge reserve and skill operation of international nursing managers, can reduce the incidence of acquired infections in hospitals, and can help the global conference to formulate relevant measures to reduce infections. Pulmonary infection is one of the most common clinical complications of laparoscopic surgery. Therefore, it is necessary to give scientific nursing measures to patients during the perioperative period, which will be helpful to the prognosis and recovery of patients. Nursing reports involving this kind of operation have been reported in previous domestic clinical reports, but they are not very specific. Based on the above research background, we found that Amour et al. reported that continuous wound perfusion under local anesthesia was effective in preventing pneumonia after sternotomy, but patients still had a certain risk of pulmonary infection [4]. Kang et al. showed that the incidence of nonventilator ICU acquired pneumonia after cardiothoracic surgery cannot be ignored [5]. Aiolfi et al. reported that laparoscopic surgery can significantly increase postoperative pneumonia and mortality in elderly patients [6]. So, it can be seen that the occurrence of pulmonary infection after laparoscopic surgery increases the difficulty of postoperative care for patients, which is one of the urgent nursing problems to be solved by nurses. The study of Obermair et al. confirmed that scientific and reasonable hospital nurse staffing can significantly improve the quality of care after pediatric laparoscopic surgery [7]. Therefore, by studying the influencing factors of pulmonary infection after laparoscopic surgery, this study aims to provide a reference basis for the development of clinical nursing programs, further achieving the goal of reducing the risk of complications and promoting the early recovery of patients. Other studies have reported that a large number of drug-resistant strains have emerged with the antibacterial drugs used widespread increasingly in clinical practice in recent years, which has also caused great trouble for the treatment of clinical infection, and even brought the loss of the best treatment opportunity for patients, leading to the aggravation of the condition and death at last [8]. Therefore, how to prevent pulmonary infection after laparoscopic surgery effectively and detect drug-resistant bacteria accurately is of great significance for the prevention and treatment of pulmonary infection. We want to investigate and analyze the risk of pulmonary infection after laparoscopic surgery and the detection results of drug-resistant bacteria. In view of this, this work studied the influencing factors of lung infection in laparoscopic surgery in the hospital and tested and analyzed its drug-resistant bacteria, in order to clarify the distribution of drug-resistant bacteria after laparoscopic surgery in hospital operating room, then choose a more reasonable and effective plan for the clinical treatment, and to provide a reference basis for the prevention and treatment of postoperative pulmonary infection at the same time; in order to improve the prognosis of patients, the following report is made.

## 2. Methods

### 2.1. Participants

Six hundred patients who received laparoscopic radical gastrectomy in our hospital from January 2017 to September 2021 were included in the study. Inclusion criteria [9] were as follows: all of them underwent selective laparoscopic radical surgery, all participants were diagnosed as gastric cancer by surgical pathology, 18 years old or more, and no infection before admission. Exclusion criteria were as follows: patients switching to open laparotomy and patients with communication disorders or accompanied by mental illness. All the included subjects signed the informed consent forms, and this study was approved by the Ethics Committee of The Second Affiliated Hospital of Qiqihar Medical University.

### 2.2. Method of Data Collection

In statistics and analysis of the overall data proportion of surgical patients in our hospital, 600 patients were selected for analysis with appropriate proportion and sufficient sample size, which was not only representative but also of high importance.

1. Pathogen detection: all patients with pulmonary infection were gargled with normal saline 2-3 times in the morning, performed aseptic operation strictly, and sputum samples from patients with deep cough were collected for examination. Sputum culture was carried out with blood agar medium, and the distribution of pathogenic bacteria was identified by an automatic pathogen identification instrument (Delica Biotechnology Co., Ltd.). The quality control strains included *Pseudomonas aeruginosa* ATCC27853, *Staphylococcus aureus* ATCC25923, *Escherichia coli* ATCC25922, *Streptococcus pneumoniae* ATCC96919, and *Klebsiella pneumoniae* ATCC28243. The above quality control strains are purchased from Baogelo Biotechnology Co., Ltd.
2. The paper diffusion method was used for the drug sensitive test, and the standard to judge the results mainly referred to the relevant standards established by the American Committee for Standardization of Clinical Laboratories in 1999.
3. Basic data collection: the demographic questionnaire was completed based on the basic data, including age, gender, smoking history, hypoproteinemia, catheterization time, diabetes mellitus, pulmonary disease history, and perioperative blood transfusion (Table 1).

### 2.3. Observation Index

To analyze the distribution of pulmonary infection in patients with laparoscopic surgery, the drug resistance of major pathogens in infectious pathogens, and the influencing factors of postoperative pulmonary infection in patients with laparoscopic surgery.

### 2.4. Evaluation Standard

The diagnostic criteria for pulmonary infection are as follows [9]: with cough, expectoration, and bubbles in the lungs and there are any one of the following: (1) the proportion of total number of white blood cells or (and) the neutrophils was significantly increased; (2) the body temperature is higher than 37.5°C; and (3) it was found in the results of X-ray that there was inflammatory infiltration in the lungs.

### 2.5. Data Analysis

Data analysis was completed with the help of SPSS 20.0 software mainly, indicated with (*n* (%)) for counting data, and the *χ*^2^ test was performed. The measurement data were expressed as ($\bar{x}\pm s$), and the *t*-test was performed. Postoperative pulmonary infection was taken as the dependent variable and hypoproteinemia, catheter insertion time, combined diabetes, history of pulmonary disease, and perioperative blood transfusion as the independent variables. Multivariate logistic regression analysis was used to analyze the risk factors of postoperative pulmonary infection in patients undergoing laparoscopic surgery. *P* < 0.05 indicated significant difference.

## 3. Results

### 3.1. Single Factor Analysis of Pulmonary Infection after Laparoscopic Surgery

The number of cases of pulmonary infection after laparoscopic surgery in 600 patients was 58, accounting for 9.67%, which was in line with the usual rates. Single factor analysis showed that all of hypoproteinemia, catheterization time, diabetes mellitus, pulmonary disease history, and perioperative blood transfusion were influencing factors of postoperative pulmonary infection in patients undergoing laparoscopic surgery (all *P* < 0.05). Therefore, we may develop nursing intervention measures for the above related factors in clinical work to reduce the risk of complications (Table 2).

### 3.2. Multiple-Factor Logistic Regression Analysis of Postoperative Pulmonary Infection in Patients with Laparoscopic Surgery

Postoperative pulmonary infection was taken as the dependent variable, while the rest were independent variables. When the value was assigned, if there were related symptoms, they were denoted as 1; if there was none, they were denoted as 0. In addition, catheterization time more than 72 h = 1, and catheterization time 72 h or less than 72 h = 0. The multifactor logistic regression analyzed that hypoproteinemia, diabetes mellitus, pulmonary disease history, and perioperative blood transfusion were all independent risk factors for postoperative pulmonary infection in patients undergoing laparoscopic surgery. These are given in Table 3.

### 3.3. Analysis on the Distribution of Pathogenic Bacteria of Pulmonary Infection after Laparoscopic Surgery

The pathogenic bacteria of pulmonary infection after laparoscopic surgery were *Klebsiella pneumoniae*, *Staphylococcus aureus*, *Pseudomonas aeruginosa*, *Escherichia coli*, and *Streptococcus pneumoniae* in order of proportion from high to low (Table 4).

### 3.4. Drug Resistance Analysis of Main Pathogenic Bacteria in Pulmonary Infection after Laparoscopic Surgery

*Klebsiella pneumoniae*, *Staphylococcus aureus*, *Pseudomonas aeruginosa*, and *Escherichia coli* have some resistance to common antimicrobial bacteria, while the resistance to vancomycin is 0.00%, 0.00%, 11.11%, and 0.00%, respectively (Table 5).

## 4. Discussion

The results of this study showed that the number of cases of pulmonary infection after laparoscopic surgery in 600 patients was 58, accounting for 9.67%. The results of Caruso et al. [10] showed that the hospital infection rate after laparoscopic surgery for gastric cancer was higher, which may be related to the fact that the study reported total hospital infections and not just lung infections. In addition, Chouhan et al. reported [11] that the incidence of pulmonary infection in elderly patients after laparoscopic radical gastrectomy was about 3%, significantly lower than that in this study, which may be caused by the small sample size of this study. Blood glucose levels are generally high in patients with diabetes mellitus, microangiopathy is often present, and the phagocytic ability of macrophages decreased in varying degrees, which decreased the immune ability of the body and finally increased the risk of pulmonary infection. All in all, patients are prone to lung infection after laparoscopic surgery, which increases the difficulty of clinical nursing work, which is worthy of clinical attention. Compared with traditional open surgery, it has advantages such as less trauma, less patients pain, and faster postoperative recovery. However, laparoscopic surgery is still one of the invasive operations, which may also cause a series of surgical complications, including incision infection, lung infection, urinary tract infection, and catheter-related infection. This study can provide very detailed data and sample support for nursing managers, help them to screen relevant cases, and make scientific and reasonable nursing research and judgment, thus contributing to the enrichment of the international health care knowledge system.

In addition, hypoproteinemia, concomitant diabetes mellitus, pulmonary disease history, and perioperative blood transfusion were the independent risk factors for pulmonary infection after laparoscopic surgery. This was highly consistent with previous studies [12, 13]. After analyzing the reasons, we believe that hypoalbuminemia may lead to the decrease of plasma osmotic pressure, which may lead to oedema of lung tissue, further cause the occurrence of pulmonary blood circulation disorder, and finally increase the risk of pulmonary infection, and hypoalbuminemia will inhibit the synthesis of immune protein to a certain extent and then promote the decrease of immune ability of the body, which is prone to pulmonary infection [14, 15]. Therefore, we should timely correct patients with hypoproteinemia, regulate the synthesis of immune proteins, and improve the immune function of patients, thus preventing the occurrence of pulmonary infection. Therefore, the perioperative and postoperative blood glucose levels should be controlled in clinical work, which may have a positive effect on the prevention of pulmonary infection. Patients with perioperative blood transfusion often have a relatively poor immune function, coupled with the influence of surgical stress, which leads to a significant decrease in immune function and is prone to postoperative infection. This suggests that we should pay more attention to perioperative patients with blood transfusion in practical work. By adjusting the diet plan and nutrition support plan, we can enhance the immune function of patients or improve the surgical or anesthesia technology to reduce the stress of surgery, so as to further avoid the occurrence of postoperative pulmonary infection. It has been confirmed that the degree of surgical trauma and stress is obvious in patients who receive blood transfusion because of acute blood loss during operation, which will inhibit their immune system, and the blood transfusion operation will aggravate the inhibition [16, 17]. Therefore, it is possible to reduce the risk of pulmonary infection by formulating relevant measures in clinical works, according to the above risk factors [18, 19].

In addition, it was found that the main pathogens of pulmonary infection after laparoscopic surgery were *Klebsiella pneumoniae*, *Staphylococcus aureus*, *Pseudomonas aeruginosa*, Escherichia *coli*, and streptococcus *pneumoniae*. The main reason may be that *Klebsiella pneumoniae* belongs to one of the normal flora of the human upper respiratory tract and intestinal tract and is a conditioned infection strain, which is easy to cause pulmonary infection when the body's resistance and immunity are reduced [20, 21]. This suggests that we should focus on the relationship between *Klebsiella pneumoniae* and pulmonary infection in clinical work and then give targeted antibiotic intervention to patients to further prevent the occurrence of pulmonary infection. In addition, *Klebsiella pneumoniae*, *Staphylococcus aureus*, *Pseudomonas aeruginosa*, and *Escherichia coli* have some resistance to common antimicrobial bacteria, while the resistance to vancomycin is 0.00%, 0.00%, 11.11%, and 0.00%, respectively. This is highly consistent with the study reported by Liu et al. [22, 23], indicating that vancomycin treatment of infections caused by *Klebsiella pneumoniae*, *Staphylococcus aureus*, *Pseudomonas aeruginosa*, and *Escherichia coli* may achieve a relatively ideal effect and is worthy of clinical promotion and application.

## 5. Conclusion

In summary, hypoproteinemia, combined with diabetes, pulmonary disease history, and perioperative blood transfusion can increase the risk of pulmonary infection after laparoscopic surgery, suggesting that in the clinical nursing process, relevant intervention measures should be formulated and implemented in accordance with the above risk factors, so as to reduce the incidence of complications and promote the recovery of patients.

The practical significance of this study lies in that the survey conclusions are representative and can provide scientific, meticulous, and extensive data support for the relevant knowledge system. Through in-depth research, it can help nursing managers to enrich their own knowledge structure, prevent and screen related cases, and make targeted nursing interventions. As for the treatment, on the basis of paying attention to pathogenic bacteria and antibacterial drugs, the new diagnostic criteria are applied to analyze the cases, so as to obtain better conclusions. However, there are still some limitations in this study. For example, the subjects included in this study are all gastric cancer patients, and no analysis has been conducted on other types of laparoscopic surgery patients, which may lead to a certain degree of bias in the research results. Therefore, it is necessary to increase the sample size in future studies to obtain more accurate and reliable data through multicenter-controlled studies. This is our future research direction.

## Figures and Tables

**Table 1:** The main contents of the demographic questionnaire.

Number	Item
1	How old are you?
2	What is your gender?
3	Do you have a smoking history?
4	Is there hypoproteinemia in your medical records?
5	How many hours of your catheterization time?
6	Does your underlying disease include diabetes?
7	Do you have a history of lung disease?
8	Did you have a blood transfusion during the operation?

**Table 2:** Single factor analysis of pulmonary infection after laparoscopic surgery.

Influencing factor		Number of cases	Infection rate	*χ* ^2^ value	*P* value
Gender	Male	357	36 (10.08)	0.176	0.675
	Female	243	22 (9.05)		
Age	≤60	378	35 (9.26)	0.194	0.659
	≥60	222	23 (10.36)		
Smoking history	Yes	217	18 (8.29)	0.733	0.392
	No	383	40 (10.44)		
Hypoproteinemia	Yes	234	37 (15.81)	16.590	0.000
	No	366	21 (5.74)		
Catheterization time (h)	>72	287	38 (13.24)	8.047	0.005
	≤72	313	20 (6.39)		
Combined diabetes	Yes	201	32 (15.92)	13.537	0.000
	No	399	26 (6.52)		
History of pulmonary disease	Yes	187	29 (15.51)	10.616	0.001
	No	413	29 (7.02)		
Perioperative blood transfusion	Yes	265	33 (12.45)	4.219	0.040
	No	335	27 (7.46)		

**Table 3:** Multiple-factor logistic regression analysis of postoperative pulmonary infection in patients with laparoscopic surgery.

Hazards	Regression coefficient	Standard error	Wald value	*P* value	OR value	95% CI
Hypoproteinemia	0.680	0.482	6.203	0.002	1.442	1.124–6.697
Catheterization time > 72 h	0.136	0.084	1.034	0.145	1.175	0.862–1.183
Combined diabetes	0.875	0.602	11.485	0.001	2.073	1.769–7.552
History of pulmonary disease	0.642	0.511	17.473	0.000	1.769	1.385–8.042
Perioperative blood transfusion	0.437	0.249	8.755	0.005	2.385	1.850–10.385
Constant term	−2.394	1.384	5.973	0.002	0.001	—

**Table 4:** Analysis on the distribution of pathogenic bacteria of pulmonary infection after laparoscopic surgery (case, %).

Nosophyte		Number of cases	Proportion (%)
Gram-negative bacteria	*Klebsiella pneumoniae*	19	32.76
	*Pseudomonas aeruginosa*	9	15.52
	*Escherichia coli*	7	12.07
Gram-positive bacteria	SA	13	22.41
	*Streptococcus pneumoniae*	5	8.62
	*Hemolytic streptococcus*	2	3.45
Fungus	*Candida albicans*	2	3.45
	Others	1	1.72

**Table 5:** Drug resistance analysis of main pathogenic bacteria in pulmonary infection after laparoscopic surgery (case, %).

Antibacterials	*Klebsiella pneumoniae* (*n* = 19)		SA (*n* = 13)		*Pseudomonas aeruginosa* (*n* = 9)		*Escherichia coli* (*n* = 7)	
	Number of drug resistant	Drug resistance rate (%)	Number of drug resistant	Drug resistance rate (%)	Number of drug resistant	Drug resistance rate (%)	Number of drug resistant	Drug resistance rate (%)
Cefazolin	8	42.11	7	53.85	9	100.00	6	85.71
Ampicillin	19	100.00	9	69.23	9	100.00	7	100.00
Ciprofloxacin	8	42.11	8	61.54	4	44.44	3	42.86
Levofloxacin	10	52.63	7	53.85	2	22.22	3	42.86
Gentamicin	8	42.11	6	46.15	4	44.44	4	57.14
Vancomycin	0	0.00	0	0.00	1	11.11	0	0.00

## Data Availability

The datasets used and/or analyzed during the current study are available from the corresponding author upon request.
